# Study on Correlation between Body Cell Mass Index and Cognitive Impairment in Hemodialysis Maintaining Patients: A Cross-Sectional Study

This article has been retracted.

**DOI:** 10.1155/2022/9023562

**Published:** 2022-03-03

**Authors:** Qinqin Ou, Chaomin Zhou, Maolu Tian, Xiangyan Yang, Yan Zha

**Affiliations:** ^1^Zunyi Medical University, Zunyi 563000, China; ^2^Department of Nephrology, Guizhou Provincial People′s Hospital, Guiyang 550002, China

## Abstract

**Objective:**

To investigate the relationship between body cell mass index (BCMI) and cognitive impairment in maintaining hemodialysis (MHD) patients.

**Methods:**

We collected the general materials, laboratory indexes, and physical measurement indexes of patients undergoing maintenance hemodialysis in hemodialysis centers of 20 tertiary and tertiary general hospitals in Guizhou Province from June to September 2020. The body composition was measured by bioelectrical impedance method, and the BCMI value was calculated. The subjects were divided into normal cognitive function group (score ≥27), mild cognitive impairment group (score 23–26), and severe cognitive impairment group (score <23). Two groups of people with normal cognitive function and cognitive impairment with similar baseline data (gender, age, and education) were obtained by propensity score matching (PSM).

**Results:**

A total of 2008 subjects were included in this study, including 467 cases (23.3%) in the cognitive impairment group. A total of 814 cases were accurately matched after PSM. Multivariate logistic regression analysis showed that the incidence risk of the BCMI Q1 group was 8.99 times higher than that of the Q4 group (95% CI: 5.74 ∼ 14.09, *P* < 0.001). ROC curve analysis showed that the best threshold of BCMI for predicting cognitive impairment in MHD patients was 9.05, the sensitivity and specificity were 71.5% and 62.7%, respectively, and the area under the curve was 0.713 (95% CI: 0.678 ∼ 0.748, *P* < 0.001).

**Conclusions:**

BCMI is related to cognitive impairment in MHD patients and has predictive value for the onset of cognitive impairment in MHD patients.

## 1. Introduction

Cognitive impairment (CI) refers to the defects of one or more key brain functions such as learning, memory, complex attention, executive function, language, perceptual motor function, and its severity can range from mild cognitive impairment (MCI) to severe dementia [1]. Maintenance hemodialysis (MHD) patients often have different degrees of cognitive impairment, and the morbidity rate is as high as 18.8%–60.9% [2–4]. Cognitive impairment can significantly increase the hospitalization rate and mortality of MHD patients and seriously affect the clinical prognosis of patients [5–7]. Therefore, it is particularly important to identify the risk factors of cognitive impairment in MHD patients as soon as possible and carry out early intervention.

Malnutrition is common in patients of maintenance hemodialysis (MHD), featuring decreased protein and energy reserves and decreased muscle mass. Studies have found that malnutrition is an important factor bringing about brain function and neurodegenerative diseases [8–12] and is closely related to the occurrence and development of cognitive dysfunction. It impacts on cognitive function in the following ways: malnutrition leads to the shortage of important micronutrients like vitamins and essential fatty acids, which is likely to stimulate the inflammation to appear in the body, and the increase in inflammatory factors and oxidative stress leads to neuroinflammation and cerebrovascular damage [8, 13]. Second, the *β*-amyloid 42 (A*β*42) drops and total tau and phosphorylated tau protein levels rise in cerebrospinal fluid (CSF) of malnourished patients, resulting in the mitochondrial dysfunction and cell death of hippocampal neurons in the brain [14, 15]. Besides energy and hormone metabolism change, and the levels of hormones related to cognitive function, like leptin, are reduced in malnourished patients [15, 16], accompanying with the decreased muscle masses that are related to the reduced volume of prefrontal, cingulate, occipitotemporal, and cerebellar gray matter [15–18].

In the current nutrition guidelines for chronic kidney disease, body mass index (BMI) is chosen as the main nutritional assessment index [19]. However, BMI values cannot differentiate between fluid, fat, and fat-free mass, the decreased muscle mass may be mistaken for increased extracellular water in MHD patients with fluid overload, and it is unable to identify the early malnutrition in MHD patients by monitoring BMI alone [20]. Body cell mass (BCM) is the key to determine the body's energy expenditure, protein requirements, and metabolism; it is a part of lean mass and does not cover extracellular water [21]. Body cell mass index (BCMI) is a BCM normalized by height. Studies have shown that the lower the BCMI, the higher the risk of death in MHD patients, and most patients die of malnutrition [22]. BCMI is linearly correlated with lean mass, positively correlated with serum albumin and blood lipids, serving as a sensitive indicator reflecting muscle wasting [23]. In patients with normal or high BMI, BCMI may be low. In case of malnutrition, especially pathological conditions like dialysis, BCMI is more accurate in assessing changes in muscle mass and protein tissue than BMI [24, 25], and is regarded the best indicator to evaluate the nutritional status in MHD patients [26].

However, whether there is a correlation between BCMI and cognitive impairment in MHD patients has not been reported at home and abroad. This study intends to explore the correlation between BCMI and cognitive impairment in MHD patients through a cross-sectional study of large samples in multiple centers and to evaluate the predictive value of BCMI on cognitive impairment in MHD patients.

## 2. Methods

### 2.1. Research Objectives

From June to September 2020, 2008 patients with maintenance hemodialysis in hemodialysis centers of 20 tertiary and tertiary general hospitals in Guizhou Province were selected. Inclusion criteria are (1) dialysis≥6 months, regular dialysis 3 times a week for 12 hours; (2) age ≥18 years; (3) all included patients had been informed to be consent with and sign the informed consent form. Exclusion criteria are (1) patients with severe liver failure, cerebrovascular disease, lung disease, and other related diseases that seriously affect patients' cognitive function; (2) those with mental illness, severe aphasia, and critical illness who cannot cooperate with the questionnaire survey; (3) serious limb defects and deformities or metal stents in the body that cannot be examined by bioelectrical impedance analysis; (4) severe infection in recent one month; (5) patients with definite diagnosis of tumor; and (6) people with alcohol dependence and psychotropic drug dependence.

### 2.2. Research Methods

General materials: the research group personnel shall issue a unified questionnaire for on-site investigation, including name, gender, age, occupation, education level, dialysis time, and mini mental state examination scale (MMSE), etc.

### 2.3. Cognitive Function Evaluation

The trained personnel of the research group will issue a unified MMSE questionnaire to all the subjects for on-site investigation. The total score of the evaluation scale is 30 points (including 10 points for orientation force, 3 points for memory, 5 points for attention and calculation, 3 points for memory, and 9 points for language ability). If the score is less than 27 points, it can be considered that there is cognitive impairment [27], of which 23–26 points are mild cognitive impairment, scores <23 were severe cognitive impairment.

### 2.4. Physical Measurement

All subjects were measured by trained personnel of the research group, including height, weight, etc., and body mass index (BMI) = weight/height^2^.

### 2.5. Measurement on Human Body Composition

Measurement was measured by bioelectrical impedance analyzer (BCM-7BJA4951, Fresenius, Germany), including body cell mass (BCM), lean tissue index (LTI), fat tissue index (FTI), water load (OH), extracellular water (ECW), muscle tissue mass (LTM), etc, and body cell mass index (BCMI) = BCM/height^2^.

### 2.6. Laboratory Indicators

Collect the laboratory indicators of the research subjects in recent 1 ∼ 3 months, including blood routine, creatinine, albumin, and other related indicators.

### 2.7. Statistical Method

SPSS 25.0 software was used for data analysis. The measurement data of normal distribution are expressed in ‾*x* ± *s*. The independent sample *t* test is used for the comparison between the two groups, and the one-way ANOVA is used for the comparison between multiple groups, the measurement data of non normal distribution are described by M (P25, p75), and Mann–Whitney U is used for comparison between the two groups, Kruskal–Wallis H test was used for multi group comparison; categorical variables were expressed by the number of cases and percentage (%), and *χ*^2^ inspection was used for inter group comparison; they are all both-side inspection according to the inspection level *α* = 0.05, when *P* ≤ 0.05, the difference was statistically significant. The caliper value was taken as 0.001 for propensity score matching (PSM). The matched data were analyzed by logistic regression analysis to analyze the relationship between BCMI and related indicators, and the risk of cognitive impairment in MHD patients and the predictive effect of BCMI on cognitive impairment were analyzed by ROC curve.

## 3. Results

### 3.1. Baseline Characteristics of Participants

A total of 2008 MHD patients were included in this study, including 1145 males (57%) and 863 females (43%), aged (53.8 ± 14.7) years, 467 patients with cognitive impairment, with a morbidity rate of 23.3%. The sickness rate of each age segment was 9.9%, 32.8%, 39.6%, and 50.6% respectively. The morbidity rate of cognitive impairment increased with age, and the sickness rate of severe cognitive impairment also increased with age (Figure 1).

### 3.2. Comparison of Clinical Characteristics between the Normal Pre PSM Cognitive Function Group and the Cognitive Impairment Group

According to the score of cognitive function, the research subjects were divided into the normal cognitive function group and the cognitive impairment group. Compared with the normal cognitive function group, the educational level, dry weight, extracellular water, lean tissue index, muscle mass, body mass index, albumin, and serum creatinine for the cognitive impairment group were lower, and there were fewer male patients for the cognitive impairment group, but age and fat tissue index for the group were higher, and the differences were statistically significant (*P* < 0.05) (Table 1).

### 3.3. Comparison of Clinical Characteristics of Different BCMI Groups before PSM

According to the three cut-off points of BCMI quartile (7.17, 8.52, 10.08), they are divided into Q1, Q2, Q3, and Q4 groups. Compared with BCMI Q2 ∼ Q4 groups, the BCMI Q1 group has fewer male patients, the highest prevalence of cognitive impairment (33.3%), higher age, dialysis age, water load, and fat tissue index, while MMSE score, predialysis BMI, postdialysis BMI, dry weight, extracellular water, lean tissue index, muscle mass, albumin, and serum creatinine were lower, the difference was statistically significant (*P* < 0.05), and there was no significant difference in hemoglobin among different BCMI groups (*P* > 0.05) (Table 2).

### 3.4. Comparison of Clinical Characteristics after PSM

In order to balance the baseline data of the two groups, taking the cognitive impairment group as the benchmark, 1:1 PSM was matched, and the caliper value was 0.001. A total of 407 pairs were successfully matched, with a total of 814 cases. There was no significant difference in gender, age, and education between the two groups (*P* > 0.05).

Comparison of clinical characteristics between patients with normal cognitive function and patients with cognitive impairment after PSM: compared with the normal cognitive function group, the cognitive impairment group had lower dry weight, extracellular water, lean tissue index, muscle mass, body mass index, albumin, and serum creatinine, but higher dialysis age, water load, and fat tissue index, all differences were statistically significant (*P* < 0.05), there was no significant difference in hemoglobin between the two groups (*P* > 0.05) (Table 3).

### 3.5. Comparison of Clinical Characteristics of Different BCMI Groups after PSM

They were divided into Q1, Q2, Q3, and Q4 groups according to the three cut-off points of BCMI quartile (7.40, 8.73 and 10.58). Compared with the BCMI Q2 ∼ Q4 groups, the BCMI Q1 group had the highest prevalence of cognitive impairment, higher age, dialysis age, water load, fat tissue index, while MMSE score, predialysis BMI, postdialysis BMI, dry weight, extracellular water, lean tissue index, muscle mass, albumin, and serum creatinine were lower, and there were fewer male patients, the difference was statistically significant (*P* < 0.05). There was no significant difference in education and hemoglobin among different BCMI groups (*P* > 0.05) (Table 4).

### 3.6. Binary Logistic Regression Analysis of the Risk of Cognitive Impairment in Patients with BCMI and MHD after PSM

In 814 patients who were successfully matched with the propensity score matching, binary logistic regression was used so as to analyze the relationship between BCMI and the risk of cognitive impairment in MHD patients. In the uncorrected model, the risk of cognitive impairment in the BCMI Q1 group was 8.992 times higher than that in the Q4 group (95% CI 3.186 ∼ 7.530 *P* < 0.05), and the risk of cognitive impairment in the BCMI Q2 and Q3 groups were 4.898 times higher than that in the Q4 group (95% CI 4.462 ∼ 13.723 *P* < 0.05), 2.620 times higher than that in the Q4 group (95% CI 1.709 ∼ 4.018 *P* < 0.05). After correcting dialysis age, creatinine, albumin, and hemoglobin, the morbidity risk of the BCMI Q1 group was 8.767 times higher than that of the Q4 group (95% CI 5.471 ∼ 14.101 *P* < 0.05), the BCMI Q2 group, and the Q3 group were 4.876 times higher than that of the Q4 group (95% CI 3.134 ∼ 7.587 *P* < 0.05) and 2.634 times higher (95% CI 1.704 ∼ 4.072 *P* < 0.05). After further correction of predialysis BMI, postdialysis BMI, OH, FTI, and ECW, the morbidity risk of the BCMI Q1 group, the Q2 group, and the Q3 group was 7.759 times (95% CI 4.421 ∼ 13.620, *P* < 0.05), 4.469 times (95% CI 2.720 ∼ 7.341, *P* < 0.05), and 2.435 times (95% CI 1.536 ∼ 3.859, *P* < 0.05) than that of the Q4 group (Table 5).

### 3.7. Binary Logistic Regression Analysis on the Morbidity Risk of Cognitive Impairment in Patients with Predialysis BMI and MHD after PSM

According to the WHO standard of BMI, the research subjects were divided into G1 (BMI < 18.5 kg/m^2^), G2 (18.5 kg/m^2^ ≤ BMI < 25.0 kg/m^2^), G3 (25.0 kg/m^2^ ≤ BMI < 30.0 kg/m^2^), and G4 (BMI ≥ 30.0 kg/m^2^). In 814 patients who were successfully matched with the propensity score matching, binary logistic regression was used so as to analyze the relationship between predialysis BMI and the risk of cognitive impairment in MHD patients. In the uncorrected model, the morbidity risk of the predialysis BMI G1 group was 2.366 times than that of the G4 group (95% CI 1.056 ∼ 5.300, *P* < 0.05). After adjusting dialysis age, creatinine, albumin, hemoglobin, and further adjusting dry weight, OH, FTI, and ECW, the correlation between predialysis BMI and the morbidity risk of cognitive impairment in MHD patients was not statistically significant (*P* > 0.05) (Table 6).

### 3.8. Binary Logistic Regression Analysis on the Morbidity Risk of Cognitive Impairment in Patients with after Dialysis BMI and MHD after PSM

According to the WHO standard of BMI, the research subjects were divided into four groups: D1 (BMI < 18.5 kg/m^2^), D2 (18.5 kg/m^2^ ≤ BMI < 25.0 kg/m^2^), D3 (25.0 kg/m^2^ ≤ BMI < 30.0 kg/m^2^), and D4 (BMI ≥ 30.0 kg/m^2^). In 814 patients who were successfully matched with the propensity score matching, binary logistic regression was used so as to analyze the relationship between after dialysis BMI and the risk of cognitive impairment in MHD patients. In the uncorrected model, the morbidity risk of BMI in the group D1 after dialysis was 3.513 times that in the group D4 (95% CI 1.419 ∼ 8.693, *P* < 0.05). After adjusting for dialysis age, creatinine, albumin, and hemoglobin, the morbidity risk of postdialysis BMI D1 group was 3.112 times higher than that of the D4 group (95% CI 1.249 ∼ 7.751, *P* < 0.05). After further adjusting for dry weight, OH, FTI, and ECW, there was no significant correlation between postdialysis BMI and the morbidity risk of cognitive dysfunction in MHD patients (*P* > 0.05) (Table 7).

### 3.9. The ROC Curve after PSM Evaluated the Predictive Value of BCMI, Predialysis BMI and Postdialysis BMI for Cognitive Impairment in MHD Patients

As shown in Figure 2, the sensitivity of BCMI for predicting cognitive impairment in MHD patients was 71.5%, the specificity was 62.7%, the optimal threshold was 9.0, and the area under the curve was 0.713 (95% CI 0.678 ∼ 0.748, *P* < 0.001). The area under the curve of BMI before dialysis and BMI after dialysis were 0.571 (95% CI 0.532 ∼ 0.610, *P* < 0.001) and 0.570 (95% CI 0.530 ∼ 0.609, *P* = 0.001), respectively. The area under the curve of BCMI predicting cognitive impairment in MHD patients was the highest.

## 4. Discussion

Studies have shown that chronic kidney disease (CKD) is an independent risk factor for cognitive dysfunction, and its impact on cognitive impairment has exceeded genetic factors, and morbidity rate is higher in maintenance hemodialysis (MHD) patients [28]. Epidemiological data at home and abroad show that the prevalence of cognitive impairment in MHD patients is as high as 18.8%–60.9% [2–4]. In this study, the prevalence of cognitive impairment in MHD patients was 23.3%, and the prevalence of cognitive impairment was significantly increased in patients aged 45 and over.

MHD patients with cognitive impairment have significantly reduced treatment compliance and quality of life and significantly increased hospitalization rate and mortality, which seriously affects the clinical prognosis of patients [5–7]. Current studies have found that cognitive impairment in MHD patients is related to a variety of factors. Malnutrition can affect energy metabolism, cerebrospinal fluid biochemistry, and brain volume [14, 16–18], which is one of the main risk factors for cognitive impairment in MHD patients. The risk of cognitive impairment in malnourished MHD patients is 20.0% higher than that in well-nourished patients [15]. Body mass index (BMI) is currently recognized as a nutritional evaluation index. However, MHD patients generally have increased water load, BMI cannot distinguish specific human components, and fluid overload in the body will cause false high BMI, thus overestimating the nutritional status of MHD patients [19, 20]. Body cell mass (BCM) is the nonfat content excluding external bone minerals and extracellular water (ECW). Body cell mass index (BCMI) refers to the ratio of BCM to height ^2^. This index does not include extracellular water (ECW), so it is not affected by body fluid changes. It is more accurate than BMI in assessing the nutritional status of MHD patients [21, 26]. The study of Talluri et al. found that when BCMI is low, it may be accompanied by decreased muscle mass and/or increased fat mass, suggesting poor nutritional status [17]. In this study, compared with the high BCMI (Q4) group, the lean tissue index and muscle mass in the low BCMI (Q1) group were significantly increased, while the fat mass index was significantly reduced, which was consistent with the study results of Talluri et al. This study also suggests that male patients may have higher BCMI values.

This study found that the dry weight, lean8 tissue index, muscle mass, and albumin in the cognitive impairment group were lower than those in the normal cognitive function group, suggesting that malnutrition is related to cognitive impairment in MHD patients. Kim et al. found that the decline of BMI is an independent risk factor for the sharp decline of cognitive function and a predictor of the progress of cognitive impairment [29, 30]. In this study, BMI before and after dialysis is related to the risk of cognitive impairment in MHD patients, but after adjusting for other risk factors, the morbidity risk of cognitive impairment in patients with BMI and MHD before and after dialysis is not statistically significant, which is different from the above research results. It is speculated that it may be related to different research objects and research methods. However, BCMI was independently associated with the morbidity risk of cognitive impairment in patients with MHD. The lower the level of BCMI, the higher the morbidity risk of cognitive impairment, the higher the prevalence. The ROC curve was further used to explore the predictive value of BCMI, predialysis BMI, and postdialysis BMI on cognitive impairment in MHD patients. The results showed that BCMI had the highest AUC for predicting cognitive impairment in MHD patients and had high predictive value for the occurrence of cognitive impairment in MHD patients. The best value for predicting cognitive impairment was 9.0, and cognitive impairment is less likely to occur when it is higher than 9.0.

In conclusion, BCMI is the influencing factor of cognitive impairment in MHD patients and has high predictive value for the occurrence of cognitive impairment. However, this study also has some limitations. First, the research objects of this study are selected from the maintenance hemodialysis center of tertiary hospitals in Guizhou Province in 2020. It is necessary to further study the patients in the dialysis center of secondary and lower hospitals. Second, this study is a cross-sectional study, which cannot reflect the causal relationship between BCMI and cognitive impairment in MHD patients. Therefore, it needs to be further verified by multicenter and large sample cohort study.

## Figures and Tables

**Figure 1:** Morbidity rate of cognitive impairment in MHD patients of different age groups.

**Figure 2:** Predictive efficacy of BCMI, predialysis BMI, and postdialysis BMI on cognitive impairment in MHD patients. Note: BCMI is body mass index, BMI is body mass index, and MHD is maintenance hemodialysis.

**Table 1:** Clinical characteristics of MHD patients with normal cognitive function and cognitive impairment before PSM.

Item	Normal cognition (*n* = 1541)	Cognitive impairment (*n* = 467)	Statistic value	*P* Value
Male [case(%)]	923(59.9)	222(47.5)	22.336	＜0.001
Age [years old, ‾*x* ± *s*]	51.44 ± 14.33	61.78 ± 13.23	−14.511	＜0.001
Educational level (below junior high school)	1034(67.1)	398(85.2)	57.557	＜0.001
Dialysis age (months)	42.90(21.00,74.95)	43.80(25.60,74.50)	−0.862	0.389
BMI before dialysis (kg/m^2^)	23.29 ± 3.69	23.25 ± 3.75	0.200	0.841
BMI after dialysis(kg/m^2^)	22.39 ± 3.63	22.44 ± 3.66	−0.248	0.804
Dry weight(kg)	58.10(51.15,66.40)	57.00(49.90,65.20)	−2.309	0.021
OH(L)	0.50(-0.50,1.60)	0.60(-0.30,1.50)	−1.116	0.264
ECW(L)	14.50(12.60,16.60)	13.90(12.00,16.00)	−3.533	＜0.001
LTI(kg/m^2^)	15.20(13.20,17.40)	14.10(12.30,15.90)	−7.26	＜0.001
FTI(kg/m^2^)	6.90(4.30,10.07)	8.20(5.45,11.00)	−4.803	＜0.001
LTM(kg)	40.10 ± 9.85	35.89 ± 9.05	8.629	＜0.001
BCMI(kg/m^2^)	8.70(7.30,10.30)	7.90(6.60,9.20)	−7.44	＜0.001
Creatinine (*μ* mol/L)	962.20(772.80,1160.90)	850.20(660.90,1039.90)	−7.229	＜0.001
Hemoglobin (g/L)	109.99 ± 19.98	108.11 ± 20.65	1.761	0.078
Albumin (g/L)	40.50 ± 4.16	39.56 ± 4.60	4.177	＜0.001

*Note.* MHD is the maintenance hemodialysis; BMI: body mass index; Oh: water load; ECW: extracellular water; FTI: fat tissue index; LTI: lean tissue index; LTM: muscle tissue mass; BCMI: body cell mass index.

**Table 2:** Comparison of clinical characteristics of MHD patients before PSM grouped by BCMI quartile.

Item	BCMI grouping				Statistic value	*P* value
	Q1 group (*n* = 504)	Q2 group (*n* = 504)	Q3 group (*n* = 504)	Q4 group (*n* = 504)		
Male [case(%)]	192(38.2)	253(50.4)	306(61.0)	394(78.5)	178.734	＜0.001
Age [years old,‾*x* ± *s*]	59.03 ± 14.66	54.44 ± 15.02	51.74 ± 14.42	50.16 ± 13.29	36.717	＜0.001
Educational level (below junior high school)	366(72.9)	343(68.3)	378(75.3)	345(68.7)	8.355	0.039
Dialysis age (months)	50.13(26.55,87.28) (30.80,86.66) (30.80,86.66)	44.13(24.14,75.09)	39.12(19.96,67.92)	37.43(19.13,65.05)	36.359	＜0.001
MMSE score (分)	26.91 ± 4.38	27.79 ± 3.35	28.21 ± 3.04	28.57 ± 2.89	21.234	＜0.001
BMI before dialysis (kg/m^2^)	22.40 ± 3.63	22.83 ± 3.43	23.26 ± 3.39	24.63 ± 3.94	35.839	＜0.001
BMI after dialysis (kg/m^2^)	21.57 ± 3.56	21.99 ± 3.39	22.34 ± 3.34	23.68 ± 3.87	33.319	＜0.001
Dry weight (kg)	54.50(48.00,62.08)	56.25(49.88,64.78)	58.35(50.80,66.73)	62.60(55.47,69.85)	139.009	＜0.001
OH (L)	0.70(-0.10,1.68)	0.50(-0.50,1.60)	0.40(-0.50,1.63)	0.30(-0.90,1.40)	31.857	＜0.001
EC (L)	12.60(11.13,14.78)	13.80(12.00,15.73)	14.70(13.00,16.43)	16.30(14.60,18.00)	377.157	＜0.001
LTI (kg/m^2^)	11.80(11.00,12.40)	14.00(13.50,14.50)	15.90(15.40,16.50)	18.70(17.80,19.80)	1723.404	＜0.001
FTI (kg/m^2^)	9.00(6.20,11.40)	7.80(5.10,10.60)	6.65(4.38,9.60)	5.30(3.00,8.50)	162.847	＜0.001
LTM (kg)	29.29 ± 5.33	36.15 ± 4.98	41.29 ± 5.94	49.74 ± 8.65	913.223	＜0.001
Creatinine (*μ* mol/L)	802.15 (647.38,946.62)	903.97 (738.85,1072.25)	979.85 (777.75,1157.98)	1113.31 (899.73,1290.90)	263.554	＜0.001
Hemoglobin (g/L)	109.05 ± 20.22	110.60 ± 19.73	109.52 ± 19.59	109.03 ± 21.01	0.670	0.571
Albumin (g/L)	39.52 ± 4.45	40.25 ± 4.35	40.54 ± 4.29	40.79 ± 3.94	8.338	＜0.001
Cognitive impairment [case(%)]	167(33.3)	123(24.5)	108(21.5)	69(13.7)	54.921	＜0.001

*Note.* MHD is the maintenance hemodialysis; BMI: body mass index; Oh: water load; ECW: extracellular water; FTI: fat tissue index; LTI: lean tissue index; LTM: muscle tissue mass; BCMI: body cell mass index.

**Table 3:** Clinical characteristics of MHD patients with normal cognitive function and cognitive impairment after PSM.

Item	Normal cognition (*n* = 407)	Cognitive impairment (*n* = 407)	Statistic value	*P* value
Male [case(%)]	206(50.6)	206(50.6)	0	1.000
Age[years old,‾*x* ± *s*]	59.85 ± 12.45	59.85 ± 12.45	0	1.000
Educational level(below junior high school)	346(85)	346(85)	0	1.000
Dialysis age (months)	40.23(20.17,68.53)	44.60(26.37,74.73)	−2.581	0.010
BMI before dialysis (kg/m^2^)	24.08 ± 3.77	23.17 ± 3.69	3.486	0.001
BMI after dialysis (kg/m^2^)	23.22 ± 3.66	22.34 ± 3.60	3.467	0.001
Dry weight (kg)	60.60(52.50,68.70)	57.10(49.90,65.00)	−3.848	＜0.001
OH (L)	0.20(−0.50,1.30)	0.60(-0.30,1.50)	−2.875	0.004
ECW (L)	15.10(13.50,17.30)	14.00(12.10,16.10)	−5.077	＜0.001
LTI (kg/m^2^)	16.50(14.50,19.00)	14.30(12.60,16.10)	−9.841	＜0.001
FTI (kg/m^2^)	6.00(3.00,9.00)	7.00(5.00,10.00)	−4.745	＜0.001
LTM (kg)	43.29 ± 10.66	36.61 ± 9.90	9.654	＜0.001
BCMI (kg/m^2^)	9.65(8.50,11.42)	8.04(6.80,9.29)	−10.53	＜0.001
Creatinine (*μ* mol/L)	913.60(758.50,1123.30)	874.00(680.00,1059.60)	−2.668	0.008
Hemoglobin (g/L)	106.54 ± 21.07	108.15 ± 20.42	−1.109	0.268
Albumin (g/L)	40.57 ± 5.03	39.67 ± 5.08	2.526	0.012

*Note.* MHD is the maintenance hemodialysis; BMI: body mass index; Oh: water load; ECW: extracellular water; FTI: fat tissue index; LTI: lean tissue index; LTM: muscle tissue mass; BCMI: body cell mass index.

**Table 4:** Comparison of clinical characteristics of MHD patients after PSM grouped by BCMI quartile.

Item	BCMI group				Statistic value	*P* value
	Q1 group (*n* = 204)	Q2 group (*n* = 203)	Q3 group (*n* = 204)	Q4 group (*n* = 203)		
Male[case(%)]	76(37.3)	88(43.3)	104(51)	144(70.9)	52.40	＜0.001
Age[years old,‾*x* ± *s*]	64.70 ± 11.48	61.12 ± 12.10	57.84 ± 12.91	55.71 ± 11.38	21.878	＜0.001
Educational level (below junior high school)	178(87.3)	172(84.7)	179(87.7)	163(80.3)	5.56	0.135
Dialysis age (months)	55.16(30.80,86.66)	38.87(25.40,72.63)	42.86(22.33,68.83)	36.17(19.10,66.50)	18.79	＜0.001
MMSE score(分)	24.25 ± 4.81	25.64 ± 4.17	26.73 ± 3.78	27.85 ± 3.32	29.23	＜0.001
BMI before dialysis (kg/m^2^)	22.41 ± 3.78	23.36 ± 3.34	23.57 ± 3.65	25.15 ± 3.73	20.05	0.001
BMI after dialysis (kg/m^2^)	21.67 ± 3.68	22.57 ± 3.32	22.68 ± 3.56	24.22 ± 3.60	18.16	＜0.001
Dry weight (kg)	54.30(46.80,62.60)	57.30(51.20,64.70)	58.70(50.90,66.80)	63.50(57.10,71.20)	77.22	＜0.001
OH (L)	0.60(-0.10,1.70)	0.60(-0.50,1.50)	0.30(−0.50,1.50)	−0.10(−1.10,1.1)	26.44	＜0.001
ECW (L)	12.9(11.20,14.8)	14.10(12.70,15.90)	14.75(13.00,17.18)	16.60(15.0,18.40)	164.97	＜0.001
LTI (kg/m^2^)	12.10(11.00,12.90)	14.30(13.80,14.90)	16.30(15.73,17.0)	19.30(18.50,20.80)	722.77	＜0.001
FTI (kg/m^2^)	9.60(7.30,12.1)	7.90(5.80,11.00)	6.05(3.73,8.67)	4.00(2.10,7.20)	167.9	＜0.001
LTM (kg)	29.80 ± 5.15	36.23 ± 4.75	42.20 ± 6.49	51.61 ± 9.21	397.26	＜0.001
Creatinine (*μ*mol/L)	806.90 (630.0,926.00)	837.00 (691.00,1008.00)	930.50 (750.84,1090.67)	1055.0 (853.60,1257.2)	88.68	＜0.001
Hemoglobin (g/L)	107.99 ± 21.17	107.23 ± 20.68	106.93 ± 19.80	107.24 ± 21.46	0.096	0.962
Albumin (g/L)	39.38 ± 4.97	39.51 ± 4.09	41.10 ± 5.55	40.49 ± 5.39	5.39	＜0.001
Cognitive impairment [case(%)]	149(73)	121(59.6)	90(44.1)	47(23.2)	112.16	＜0.001

*Note.* MHD is the maintenance hemodialysis; BMI: body mass index; Oh: water load; ECW: extracellular water; FTI: fat tissue index; LTI: lean tissue index; LTM: muscle tissue mass; BCMI: body cell mass index.

**Table 5:** Correlation between BCMI and morbidity risk of cognitive impairment by binary logistic regression analysis.

Grouping	Model 1		Model 2		Model 3	
	OR (95%CI)	*P* value	OR (95%CI)	*P* value	OR (95%CI)	*P* value
BCMI Q1	8.992(5.466∼14.064)	＜0.001	8.767(5.471∼14.101)	＜0.001	7.759(4.421∼13.620)	＜0.001
BCMI Q2	4.874(3.133∼ 7.581)	＜0.001	4.876(3.134∼7.587)	＜0.001	4.469(2.720∼7.341)	＜0.001
BCMI Q3	2.620(1.709∼4.018)	＜0.001	2.634(1.704∼4.072)	＜0.001	2.435(1.536∼3.859)	＜0.001
Reference	Reference	Reference	Reference	Reference	Reference	Reference

*Note.* (1) Model 1 is an uncorrected model; (2) Model 2 was the model after correcting dialysis age, creatinine, albumin, and hemoglobin; (3) Model 3 is the model after correcting dialysis age, creatinine, albumin, hemoglobin, predialysis BMI, postdialysis BMI, dry weight, OH, FTI, and ECW.

**Table 6:** Correlation between BMI before dialysis and morbidity risk of cognitive impairment by binary logistic regression analysis.

Grouping	Model 1		Model 2		Model 3	
	OR (95%CI)	*P* value	OR (95%CI)	*P* value	OR (95%CI)	*P* value
BMI G1	2.366(1.056 ∼5.300)	0.036	2.027(0.893∼4.601)	0.091	1.155(0.434∼3.072)	0.773
BMI G2	1.586(0.874∼2.877)	0.129	1.558(0.856∼2.837)	0.147	1.349(0.669∼2.719)	0.403
BMI G3	1.119(0.594∼2.110)	0.728	1.103(0.582∼2.088)	0.764	1.081(0.539∼2.170)	0.826
Reference	Reference	Reference	Reference	Reference	Reference	Reference

*Note.* (1) Model 1 is an uncorrected model; (2) Model 2 was the model after correcting dialysis age, creatinine, albumin, and hemoglobin; (3) Model 3 was the model after correcting dialysis age, creatinine, albumin, hemoglobin, dry weight, OH, FTI, and ECW.

**Table 7:** Correlation between BMI after dialysis and the morbidity risk of cognitive impairment by binary logistic regression analysis.

Grouping	Model 1		Model 2		Model 3	
	OR (95%CI)	*P* value	OR (95%CI)	*P* value	OR (95%CI)	*P* value
BMI D1	3.513(1.419∼8.693)	0.007	3.112(1.248∼7.760)	0.015	1.155(0.434∼3.072)	0.773
BMI D2	2.23(0.998∼4.984)	0.051	2.172(0.968∼4.876)	0.06	1.349(0.669∼2.719)	0.403
BMI D3	1.997(0.854∼4.670)	0.11	1.946(0.828∼4.571)	0.127	1.081(0.539∼2.170)	0.826
Reference	Reference	Reference	Reference	Reference	Reference	Reference

*Note.* (1) Model 1 is an uncorrected model; (2) Model 2 was the model after adjusting dialysis age, creatinine, albumin, and hemoglobin; (3) Model 3 was the model after adjusting dialysis age, creatinine, albumin, dry weight, OH, FTI, and ECW.

## Data Availability

The data used to support the findings of this paper are available from the corresponding author upon request.
